# An Analysis of Students' Work Values Education Strategies and Environment Based on Psychological Contract

This article has been retracted.

**DOI:** 10.1155/2022/4798768

**Published:** 2022-08-31

**Authors:** Wujun Dai

**Affiliations:** Foshan Science and Tecnology College, Foshan 528225, China

## Abstract

An implicit agreement between people and organizations is known as a psychological contract. It represents what each party anticipates from the other in terms of giving and receiving. The psychological contract theory has forced ideological and political educators to adapt their ideas and develop new teaching strategies. The psychological expectations of the educatees can be fully mobilized and the value orientation of both sides tends to be consistent through the creation of a strong psychological contract between the educators on both sides, which will help to increase the efficacy of ideological and political education. There is theoretical and empirical support for the organizational remedy after a psychological contract breach. Student work is intended to meet the individual needs of students or the needs of society, resulting in two completely distinct values, namely, values based on individuals and values based on societies. Students' work in the new era should be a harmonious blend of personal values and social values. In the study, students' work values fluctuated about 70% of the time, and psychological contracts had a significant impact on those work values. In the past 50 years, the psychological contract theory has seen the development and refinement of its theoretical framework, the clear definition of its content and organizational principles, the behavior research following psychological contract rupture and breach, the establishment and compensation of psychological contracts, and more. The process of organization management has benefited from the continuous concretization and expansion of its application field as a management theory and method.

## 1. Introduction

A psychological contract is an understanding of the obligations and expectations between organizations and students. In recent years, the psychological contract theory has been guided, gradually demonstrating its special benefits in organizational management and education, drawing an increasing amount of attention. The values of students' work are reflected in the consciousness of others. The value relationship between the objective characteristics of students' work and the needs of the subject is reflected in people's systematic understanding and fundamental perspective of the value function of student work. The dynamics of the psychological contract and the erosion of employee loyalty, as well as the detrimental effects of a psychological breach on workers' work attitudes, work behaviors, and productivity efficiency, are the main topics of a significant body of literature research on this topic. The organizational remedy after a psychological contract breach, however, has received little attention from theoretical research and empirical evidence. Businesses across the world are dealing with more intense competition as a result of the growth of the economy and the acceleration of globalization. Many businesses must make significant changes to their business strategies and operating models to survive and advance in the market. These changes may include organizational mergers, reorganizations, layoffs, cost-cutting measures, and the implementation of new management techniques. In the growth of the global economy, the past ten years have been a turning point. As economic globalization has been gradually accelerated, strategic alliance, business expansion, merger, and reorganization strategies have undergone significant changes. These changes have also significantly altered the organizational structure of businesses. The study of psychological contract rupture is a new area of study that is becoming increasingly popular in management psychology and human resource management [1]. College students' work is characterized by two entirely different values, namely, the values centered on individuals and the values centered on society, depending on whether they are working to meet their own personal needs or the needs of society. A psychological contract is a set of expectations that an organization and its members have for one another based on their respective internal needs. Actually, a psychological contract combines the knowledge and expectations of each party regarding the duties and commitments of the other party. The psychological contract is created when both parties believe that the other party has fulfilled their duties and commitments in a manner that is consistent with either their own expectations or the initial promise made by the other party. When the psychological contract is inconsistent with the initial expectations of both parties or the gap is too wide, it is challenging to form or break if the other party breaks its psychological promise or fails to fulfill it for some reason. Through the regulation of mutual expectation and psychological contract, the introduction of psychological contract into ideological and political education enables both parties to reach a psychological consensus and fully mobilize the educated's subjective initiative, which is conducive to further improving the teaching effectiveness of ideological and political education [2, 3].

Although psychological breach of contract is common, particularly in organizations that are changing, this does not mean that businesses should disregard it. The main components of the psychological contract remedy, as well as the key for organizations to reduce the negative effects caused by the breach, are how to attribute the breach phenomenon, how to ease the students' anxiety, and how to steer the relationship between the two sides to develop in a positive direction. According to this value perspective, student work should follow the natural law of human development, take into account individual differences in development, and cultivate individuals with free development. It should also promote the free development of students' personalities. It stems from a perspective on education that emphasizes individual values. Students anticipate a positive learning environment, top-notch instructors, and an affordable talent development program from their school. The school has high standards for its students, including moral excellence, academic excellence, and a sense of social responsibility. The idea of a psychological contract is used to emphasize that, in addition to the terms set forth in a formal employment contract, there may also be implicit, informal, and undisclosed mutual expectations that play a significant role in influencing how employees behave. As a result, it is one of the crucial research areas in organizational behavior and human resource management.

In this paper, many research methods are used to further understand and explain it. In the research of the psychological contract, this paper uses the methods of establishing model diagrams and formulas to demonstrate and explain it. In the study of students' work values, a data map is established to analyze it.

The main contributions of this paper are the following:

1. Multievidence method is used to further supplement and explain its research
2. The corresponding formulas and model diagrams are established, which can be further analyzed and explained
3. The contribution of this paper is that psychological contract plays a leading role in students' work values through its research

The rest of this paper is arranged as follows: The second part introduces and discusses the related work and further discusses its research. The third part studies and explains the psychological contract. The fourth part introduces and analyzes the research on students' work values. The fifth part summarizes the full text.

## 2. Related Work

The concept of psychological contracts is becoming more and more accurate, and the lines separating the contracting parties are becoming finer as psychological contract research progresses. The subjective expectations of both educators in ideological and political teaching activities come from real life, according to the psychological contract theory. Following employees' cognitive evaluation of the organization's fulfillment of the psychological contract, some experts believe that psychological contract violation is not only cognitive but also a type of mental accumulation and emotional experience. Ideological and political education can be made more relevant and efficient by combining the psychological contract theory with it. This will allow us to analyze the crucial role that psychological contracts play in ideological and political education from the perspective of social psychology. Due to its operability, the chivalrous definition of psychological contract is simple to quantify. As a result, many institutions that conduct empirical research use it. The psychological contract is an innovation in the theory of ideological and political education for college students that begins by addressing the internal psychological needs of schools and students. It is also the physical manifestation of the humanization and rationalization of ideological and political work.

In the research, the authors think that the organization is actually a special group established by relationships [4]. When an enterprise adjusts its organizational structure and changes its employment relationship, the core element that can reflect this change is the psychological contract. George believes that the connotation of psychological contract is actually an implicit agreement between individuals and organizations [5]. Puente believes that psychological contract destruction is a cognitive change caused by employees' failure to fulfill their commitments or responsibilities in the psychological contract to the organization. That is to say, when employees realize that, in fact, they did not get what their organization promised in the past, a psychological contract breach was thus produced [6]. Li and Yang think that psychological contract damage can and does occur when there is no factual damage [7]. Lan and Mo think that the psychological contract rupture is an individual's cognition that the organization fails to fulfill one or more obligations in the individual psychological contract in a way equal to the individual's contribution [8]. Freese and Schalk think that a psychological contract can be defined as “the understanding and perception of the obligations and responsibilities contained in the relationship by both parties of the employment relationship, that is, the organization and the individual” [9]. Eckerd et al. believe that psychological contract rupture and psychological contract breach are two completely different concepts [10]. Wei et al. believe that the difference between rupture and breach is not reflected in the time sequence, nor in the difference between cognitive evaluation and emotional response, but in the recognition of the content and degree of the other party's contract performance by the relationship subject [11]. Blaevska-Stoilkovska believes that a psychological contract rupture can be equated with a psychological contract breach, both of which contain cognitive and emotional responses [12]. Zhao and Zhang Inspirational believe that the intentional breach of contract, inability to honor, and the inconsistent understanding of commitments or responsibilities between the two parties to the contract are the three main reasons for the destruction of a psychological contract [13]. In the research, Chen College proposed that psychological contract breach and psychological contract breach are two completely different concepts [14].

## 3. Psychological Contract Research and Analysis

### 3.1. Concept of Psychological Contract and Remedial Procedure

A psychological contract is the understanding and views of both parties of the employment relationship on the obligations and responsibilities contained in the relationship. The concept of the psychological contract was not taken seriously by academic circles in its early stage. Psychological contract rupture is the result of a psychological comparison between the promise of the organization and its actual income, and it is a cognitive evaluation of the content and degree of contract performance. Psychological contracts can be basically divided into two categories: transactional psychological contracts and relational psychological contracts. Breach of the psychological contract not only causes emotional harm to employees but also is very harmful to enterprises. When the organization needs employees to work more flexibly and harder, many employees retreat from the benign interactive relationship between the two sides and make negative reactions to the breach of the psychological contract, such as reevaluating the contract, reducing trust in the organization, and lowering personal performance, thus directly damaging the performance of the organization. With the development of society and the economy, education is more important to serve the economy, so the value of education in the economy is becoming increasingly obvious. Flexible management is put forward relative to rigid management. Rigid management mainly refers to such a management form that a school formulates a series of school rules and disciplines that restrict students' study, life, and practice according to existing laws and regulations. Depending on the nature of the organization, the psychological contract's content is typically broken down into two parts: the organization's obligations and responsibilities and the obligations and responsibilities of its members. Focus, from the pursuit of material and external needs to the pursuit of social and emotional needs; Duration, from the pursuit of short-term obligations and responsibilities to the pursuit of long-term or even indefinite interests; and Form and Stability of Work, from the pursuit of static and stable responsibilities to dynamic and flexible responsibilities. According to empirical research on psychological contracts in organizations, a psychological contract is an agreement between an employer and employee regarding what they should give and receive simultaneously. The implied mutual responsibility between employers and employees is the fundamental tenet of the agreement [15, 16]. Organizations are unable to keep their initial commitments to employees due to unpredictability or uncontrollability in economic and environmental factors, which also results in the abolition of psychological contracts. Providing job content, job richness and flexibility, fair compensation, opportunities for growth and promotion, adequate tools and resources, a high-quality working environment, appealing welfare, etc. are the main organizational responsibilities and obligations. The organizational setting, the workplace environment, and the psychological contract's contents all differ, and as a result, so do the psychological contract's structural elements, which primarily include two-dimensional, three-dimensional, and multidimensional elements. In the research, a model diagram is established for analysis and explanation, as shown in Figures 1 and 2.

When the two sides of the contract have different understandings of the commitments or responsibilities in the contract, psychological contract destruction will also occur. Before employees are hired, they lack sufficient communication with the organization, which leads to differences in the understanding of the employment agreement between the two parties. The greater the difference, the greater the possibility of psychological contract destruction. The psychological contract refers to a series of mutual psychological expectations, which are mutually perceived but not explicitly expressed by both parties to the contract. The two researchers emphasized “psychological expectations,” clearly put forward the specific expectations of employees and organizations for each other, and pointed out in detail which specific aspects of psychological contract can be used to motivate employees for enterprises or organizations. The formed psychological contract needs to be maintained by both contracting parties. When one or both parties realize that the psychological contract is about to break or has broken, they should take remedial measures, that is, the remedy of the psychological contract [17]. The psychological contract remedy refers to a series of compensatory actions taken when it is found that the established psychological contract may or has been broken. According to the research, the corresponding statistical data are analyzed, such as those in Tables 1 and 2.

### 3.2. Research and Analysis on the Application of Psychological Contract

The application research of psychological contract theory begins with the research on the perception, emotional response [18], and corresponding behavioral response of the fulfillment degree of responsibilities and obligations between the organization and its members. Job satisfaction of members is one of the important quality indicators of organizational management efficiency. The job satisfaction level is a common problem between organizations and members. There is a significant correlation between psychological contracts between organizations and members and job satisfaction, and job satisfaction can positively predict psychological contracts. The core of flexibility management is “people-oriented.” Its basic meaning refers to a kind of management form in which people's psychological and behavioral laws are studied, and noncoercive methods are adopted to produce potential persuasive power, influence, and driving force in people's minds, so as to turn organizational well into people's conscious actions. With the maturity of psychological contract theory and the deepening of applied research, the applied research of psychological contract has made the following breakthroughs. Since the study of the psychological contract began to enter the field of management, western researchers have described, explained, and evaluated psychological contracts from different backgrounds or angles and put forward many different theories. The construction of psychological contracts will greatly enhance the educated's learning subject status, make the educated feel respect from the organization, and improve their satisfaction with the organization. With the rapid popularization of the Internet, people can easily obtain the latest information resources in the world. This information is full of bad information, which affects people's ideology virtually. In particular, western culture has flooded into the domestic market with movies, TV, and Internet as carriers, which has exerted a subtle influence on people's traditional values. These theories are based on the characteristics of western employees and organizations and their relationship with the external environment, and they are of great reference to the study of psychological contract management in China. However, it should be noted that in the process of localization of psychological contract management research in China, the characteristics of employees and organizations in Chinese enterprises and the internal and external factors of the emergence and establishment of psychological contracts are important to the construction of localization research. In the research of psychological contract application, an algorithm formula is established to explain it, such as

(1) $$\begin{array}{c} f+\arctan\;z/2\times 1^{1}, \end{array}$$

(2) $$\begin{array}{c} \bar{f_{1}}\cdot 1\vee 2^{1}i^{\prime }<x{\left(l_{2}^{\prime }+t_{\psi }=\right)}_{u}^{x}\cdot 11, \end{array}$$

(3) $$\begin{array}{c} F_{u}+I^{\prime l}=\log\;x_{-}^{\prime \prime }C_{111}^{\infty }, \end{array}$$

(4) $$\begin{array}{c} x_{-}^{-\left(T/L_{-}^{\prime \prime }\right)\bar{y^{5}}},{\bar{t}}_{-}^{-\lambda },\frac{2}{x_{J}^{1}}+1\frac{x+1}{k}, \end{array}$$

(5) $$\begin{array}{c} \rho_{\nu }={\sum_{+1/1}^{x-1}1=\frac{\varkappa }{\mathrm{17}}\backslash \frac{1}{\Gamma }|}_{1}\cdot \pi^{lF}. \end{array}$$

One of the most intricate threads in psychological contract research is the measurement of psychological contracts. The psychological contract is based on the idea that flexible management promotes “thinking about students' needs and thinking about students' thoughts.” It can meet students' reasonable expectations, enable students to agree with the school on values and development goals, and inspire students' inner potential and subjective initiative from the bottom of their hearts by constantly understanding their needs in all areas. It is first introduced in the management field, highlighting the fact that, in addition to the formal economic expectations set forth in the relationship between individuals and organizations, there are implicit, unstated, and covert mutual psychological expectations that play a significant role in determining individual attitudes and behaviors. Different organizational environments have different interpretations of what the psychological contract means, and an inadequate understanding of concepts results in inadequate validity of quantitative research. These factors together cause different understandings of the psychological contract's connotation. The factors that affect psychological contracts can be separated into external factors from organizations or social environments and internal factors from individuals from a horizontal perspective using organizations as the dividing line.

The psychological contract is influenced by the social environment, information provided by organizations, and social clues. Because individuals are in a specific social culture and social norms, employees constantly receive information from outside and inside the organization in the process of socialization, and the psychological contract formed on this basis is bound to be influenced by this information. Ideological and political education is not just preaching but should run through the growth and success of the educated. Students' expectations of career planning and psychological contract are basically the same, and they will determine different goals, tasks, and realization paths according to their own reality. Therefore, ideological and political educators should implement classified management according to the career planning path of educational objects and try to create conditions for them to meet their different needs. In the process of constructing psychological contracts, teachers and students may use different forms of psychological suggestion to influence each other, but there are obviously individual differences in suggestion skills and comprehension ability [19, 20]. At this time, the ideological and political educators should play a more leading role, change the suggestive methods in time according to the individual differences of different educatees, and make appropriate use of language, expressions, actions, and other ways to help the educatees understand the correct meaning of suggestion, so as to make corresponding responses. Violation can reduce employees' loyalty to employers and satisfaction with work and organization and reduce the image of retention and sense of responsibility to the organization. However, these views ignore the constructive role brought by the break or breach of the psychological contract. In the research, the corresponding calculation formulas are established, such as

(6) $$\begin{array}{c} f^{\prime }=11\lambda_{y-1\cap_{=}\bar{F}}^{\left(x+L_{t/111}/2-1i\right)1}, \end{array}$$

(7) $$\begin{array}{c} 1:l_{+}^{\left(1/x\right)71^{1}}tr/\Delta_{2}^{i_{-}^{lt}\times 21}=1-1\pi +1^{\prime }, \end{array}$$

(8) $$\begin{array}{c} F_{\lambda }t_{1-t_{{\overset{⟶}{l}}^{1}}^{-A\sqrt[{ℵ}]{,1}}\Sigma }^{-0}, \end{array}$$

(9) $$\begin{array}{c} \bar{1-x}=7+\left(1\sum_{x_{-},1}^{x-1}i=7\right)-1,2^{1}, \end{array}$$

(10) $$\begin{array}{c} xctgth^{p}\frac{\pi_{-}^{\prime \prime }\lambda }{+17\cdot 1^{\Gamma }}\cdot 7. \end{array}$$

In view of the related research on psychological contract destruction, the author consulted the related literature and found that researchers have done a lot of research on the causes and consequences of psychological contract destruction but little research on the formation mechanism of the destruction. The psychological contract exists not only between individuals and groups but also between individuals and groups. For example, communication between friends is also based on a good psychological contract, based on responsibility and implicit commitment. The factors that influence psychological contracts include psychological coding, personal factors, and personality characteristics. Due to the differences in personality and ability of individual employees, they have different levels of cognitive processing, and naturally, there are some differences in their understanding of organizational information. Many researchers have studied the influencing factors, functions, and mechanisms of psychological contracts from different application fields and scenarios and have obtained certain research results. Application is the main trend of current research and should be strengthened. Applying psychological contract theory to solve practical problems in different situations and fields is the trend of future research. In various fields, although there are many applied studies, they are not deep enough on the whole, and most of them are introductory and explanatory articles, including some empirical studies, which mainly discuss the influence of psychological contract, the correlation and difference between factors, and a few experimental studies. The research of psychological contracts generally focuses on two fields. Part of the research focuses on the changes in psychological contract content, while the other part focuses on the breach of psychological contract and its negative impact on employees' attitudes and behaviors. The content of psychological contracts varies with the times. In the past, when the external environment was relatively stable and the requirements for knowledge were not high, the psychological contract paid more attention to stability, persistence, and loyalty, and the expectation for employers was to provide continuity, job stability, training, and career development. In today's unpredictable external environment and ever-increasing demand for knowledge, psychological contract emphasizes internal harmony, innovation, adaptability, and extraordinary performance, and the expectation of employers is a fair reward for new profits. On the basis of deconstructing the concept of psychological contract breach, this paper puts forward the development model of psychological contract breach, which is mainly composed of several processes, from the inability to fulfill, breaking promises, and understanding ambiguity to the perception that promises are not fulfilled, and then the psychological contract breaks down. This model points out that the organization's intentional breach of contract, inability to honor, and the two parties' inconsistent understanding of commitments or responsibilities are the three main causes of psychological contract destruction. At the beginning of the research on psychological contract rupture, the concepts of psychological contract rupture and psychological contract breach were recognized equally. With the deepening of research, rupture and breach are gradually distinguished and compared.

## 4. Research on Students' Work Values

### 4.1. Research on Work Values

Whether it is the destruction of organizational property or the failure to work, it is only the deviation behavior at the organizational level. However, in the workplace, apart from the property of the organization and the work itself, the members of the organization are actually part of the workplace environment. In the workplace environment, in addition to organizational property and work, employees' deviant behavior goals should also include interpersonal deviant behaviors, such as individuals may have verbal or physical communication and interaction with other members of the organization. When these ways violate the organization norms or hurt the members of the organization, they constitute workplace deviant behaviors referred to in the study. Values will affect the process of individual perception and then make people's perception of external stimuli consistent with their value structure. At present, the measurement of psychological contract is mainly based on scale measurement, while the compilation of scale mainly uses factor analysis and overreliance on statistical methods and neglects other methods such as classification according to actual situations. Many scholars emphasize that a psychological contract should be considered from the perspective of contracting parties, not just employees or members of organizations, so as to truly reflect the original intention of the psychological contract. Work values include a series of concepts from professional ethics to work orientation, including work orientation, work needs, and professional ethics system. It is an internal ideological system that directly affects behavior and is essentially different from external systems such as rules and regulations and legal discipline. In recent years, the psychological contract has become a hot issue in the research field of international human resources and organizational behavior. At present, there are many theoretical discussions on psychological contracts, but there are no empirical studies in some cognitive fields. Researchers' research on psychological contract destruction is mostly confined to the responsibility of employers or employees, and the field of influencing factors of psychological contract destruction needs to be expanded. As far as the employment of enterprises is concerned, if the factors of work values are taken into account when recruiting new employees, the candidates can be effectively screened, and the potential turnover rate can be reduced by recruiting employees who can correctly understand the expectations of employers, have correct values orientation, and easily establish mutual trust with the organization. In enterprise training, if employees are educated according to work values, and the collective-oriented style and behavior are strongly encouraged, the negative cognition of job seekers about organization and work can be reduced, and the turnover rate of employees in the future can be reduced. Therefore, the corresponding data graphs are established to analyze it, as shown in Figures 3–5.

In the process of socialization, people will be attracted by the benefits provided by the organization, hoping to enter and stay in the organization. At this time, individuals will show some behaviors beneficial to the organization in order to achieve this goal and consolidate their relationship with the organization. And if the organization can no longer provide benefits for the individual, then the individual will be reluctant to pay for the organization. To some extent, the implementation of workplace deviation behavior can make employees repair the psychological imbalance caused by the organization, such as employees' continuous destructive behavior and abuse of organizational resources to increase the cost of the organization, so as to balance the cost paid by the organization with that paid by employees. Psychology holds that work values are a more basic component than interest in the whole psychological structure and one of the most important components of the whole outlook on life and values.

### 4.2. Students' Work Values and Educational Analysis

Social values emphasize that a school is a tool whose purpose is to serve the politics, economy, and culture of society by cultivating the talents needed by society. Higher education in classical universities such as Oxford and Cambridge in England has itself become a manifestation of personal value, and universities basically cultivate “gentlemen” who are divorced from social reality. In the United States, it is easy for students to enjoy greater freedom in choosing disciplines and courses and teaching management. Students can choose and receive education according to their own interests, hobbies, and social needs, so as to give full play to their abilities, cultivate their independence and creativity, meet the development and perfection of individuals in free competition, and thus realize the needs of personal value. The gradual implementation of the complete credit system in colleges and universities embodies the educational concept of “people-oriented, teaching students in accordance with their aptitude,” which is conducive to the cultivation of innovative and compound talents with high quality. With the establishment of the socialist market economic system and the deepening reform of the higher education system, and the increasingly obvious tendency of logistics in higher education institutions, while bringing great changes to students' learning styles and lifestyle, students begin to question the discipline constraints of the school, and even contradictions and disputes exist objectively, which brings new challenges to the management of higher education institutions. Social-based values require that the content of students' work is mainly ideological and political work. New educational values require that the content of students' work be expanded from political work to comprehensive services for students, such as psychological counseling, employment guidance, cultural and sports activities, social practice, dormitory management, guidance on marriage and love, rights and interests protection, reward and punishment management, work-study program, and financial assistance. According to the research, a data chart is established for analysis and interpretation, as shown in Figures 6 and 7.

Student work cadres must also be transferred to different institutions after the reconstruction of student work institutions. Student work is greatly impacted by the division and divergence of student institutions and personnel. Instead of being a “handyman” and “temporary worker,” it enables the student staff to really have a professional direction. It also allows for the recruitment of more highly educated professionals to work on student projects, realizing the specialization of student work. Following their adjustment period as freshmen, students start to focus more on their future career development as their grades rise and they gradually acquire the necessary professional knowledge. Students can more easily choose training courses based on their current situation and personal interests, which will improve their practical operation ability and lay the groundwork for entering society by defining their career goals as early as possible, developing their professional awareness, and establishing their employment concept. Currently, it is widely accepted that education is valuable when it aids in social and economic construction. No error has been made. The flaw is that it ignores the demands of personal growth and the cultivation and development of personality while emphasizing the setting of training standards and designing the higher education training process in accordance with societal needs. The debate over the fundamental purposes of education has grown since the late 1980s when it was questioned whether education should be driven by the value of social development or aimed at people's self-development and self-realization. The conclusion of the argument is that people's development and social development are dialectically unified, with people's development serving as the predicate and basis for social development and as the condition and end goal of social development. The old work system cannot possibly complete the new task of student work given the development of society and the shift in people's educational values; therefore, it requires a thorough reform. The student work system needs to be rebuilt so that the student work reflects the harmony of social and personal values.

## 5. Conclusion

Cross-cultural comparative research on psychological contract breaches should be an important research direction in the future. There has been little research on the role and status of individual differences in the dynamic development of psychological contracts. However, individual differences, such as organizational justice and personality traits, play an important role in the formation and destruction of psychological contracts, which will have a potential impact on the development of the relationship between employees and organizations. When conducting direct dialogue with parents or indirect communication such as mail and telephone, schools need to help parents to establish a correct educational view, communicate with students more, and gradually form a dialogue context of equality, harmony, and mutual trust. They should treat college students as adults and social people, advocate encouraging education, appreciate their children with an appreciative attitude, give them trust, form a powerful driving force for their progress, and promote their growth by establishing psychological contracts. The psychological contract is dynamic, and it is constantly destroyed and reformed. In constant change and modification, the psychological contract of employees is becoming more and more complicated. Slight environmental turbulence may lead to the breach or even destruction of employees' psychological contracts, which is inevitable, and the organization need not worry about it.

## Figures and Tables

**Figure 1:** Model diagram of psychological contract process (1).

**Figure 2:** Model diagram of psychological contract process (2).

**Figure 3:** Data map of work values.

**Figure 4:** Data map of work value research.

**Figure 5:** Data research chart of various aspects of work value.

**Figure 6:** Data analysis of students' values (1).

**Figure 7:** Data analysis of students' values (2).

**Table 1:** Psychological contract data analysis (1).

Statistics of psychological contract data		
Category	Influence degree	Existence degree
Student	76.3%	87.3%
Staff	45.7%	45.3%
Worker	53.4%	65.3%

**Table 2:** Psychological contract data analysis (2).

Statistics of psychological contract data		
Category	Influence degree	Existence degree
Social personnel	23.4%	32.3%
Administrative staff	34.5%	23.3%
Migrant worker	53.4%	65.3%

## Data Availability

The data used to support the findings of this study are included within the article.
